# Targeting VEGFR-3/-2 signaling pathways with AD0157: a potential strategy against tumor-associated lymphangiogenesis and lymphatic metastases

**DOI:** 10.1186/s13045-017-0484-1

**Published:** 2017-06-19

**Authors:** Melissa García-Caballero, Jenny Paupert, Silvia Blacher, Maureen Van de Velde, Ana Rodríguez Quesada, Miguel Angel Medina, Agnès Noël

**Affiliations:** 1 Laboratory of Tumor and Developmental Biology, Groupe Interdisciplinaire de Génoprotéomique Appliqué-Cancer (GIGA-Cancer), Tower of Pathology, University of Liège, B23, +4, Avenue de l’hopital, 1, Sart Tilman, B-4000 Liège, Belgium; 2 Departamento de Biología Molecular y Bioquímica, Facultad de Ciencias, and IBIMA (Biomedical Research Institute of Málaga), Universidad de Málaga, Andalucía Tech, Málaga, Spain; 3 Unidad 741 de CIBER “de Enfermedades Raras”, E-29071 Málaga, Spain

**Keywords:** AD0157, Lymphangiogenesis, VEGFR-3/-2, Lymph nodes, Lymphatic metastasis

## Abstract

**Background:**

Lymphatic metastasis is one of the leading causes of death in patients with different types of cancer and is the main prognostic factor for the disease survival. The formation of new lymphatic vessels (lymphangiogenesis) in primary tumors facilitates tumor cell dissemination to regional lymph nodes and correlates with distant metastases. Lymphangiogenesis has thus emerged as a suitable therapeutic target to block metastases, but no anti-lymphangiogenic compounds have been approved for clinical use to date. Therefore, new or improved therapies blocking lymphatic metastases are urgently required.

**Methods:**

We established murine breast tumors to assess the effect of AD0157 on tumor growth, lymphangiogenesis, and lymphatic dissemination. Then, a battery of in vivo (mouse corneal neovascularization and ear sponges), ex vivo (mouse lymphatic rings and rat mesentery explants), and in vitro (proliferation, tubulogenesis, wound-healing, Boyden chambers, and spheroids) assays was used to give insight into the lymphangiogenic steps affected by AD0157. Finally, we investigated the molecular pathways controlled by this drug.

**Results:**

AD0157 was found to inhibit the growth of human breast cancer xenografts in mice, to strongly reduce tumor-associated lymphangiogenesis and to block metastatic dissemination to both lymph nodes and distant organs. The high anti-lymphangiogenic potency of AD0157 was further supported by its inhibitory activity at low micromolar range in two in vivo pathological models and in two ex vivo assays. In addition, AD0157 inhibited lymphatic endothelial cell proliferation, migration and invasion, cellular sprouting, and tube formation. Mechanistically, this compound induced apoptosis in lymphatic endothelial cells and decreased VEGFR-3/-2, ERK1/2, and Akt phosphorylations.

**Conclusions:**

These findings demonstrate the suitability of AD0157 to suppress tumor-associated lymphangiogenesis. Beyond discovering a new potent anti-lymphangiogenic drug that is worth considering in future clinical settings, our study supports the interest of designing anti-lymphangiogenic therapies to avoid distant metastatic processes.

**Electronic supplementary material:**

The online version of this article (doi:10.1186/s13045-017-0484-1) contains supplementary material, which is available to authorized users.

## Background

The elevated mortality rates seen in cancer patients are associated with the metastatic spread of tumor cells from their initial origin sites to distant tissues [1]. Although metastatic dissemination can occur via a variety of mechanisms, most metastases arise following cell intravasation into blood and/or lymphatic vasculature to further gain access to the systemic circulation [2]. Indeed, clinicopathological studies in micrometastases, frequently in breast cancers, suggest that lymphatic vessels are preferentially used as the initial route for the tumor invasion rather than blood vessels [3, 4]. This fact can be explained by the morphological advantages and structural features of lymphatic vessels that facilitate the intravasation and extravasation of tumor cells and favor their survival in the lymphatic system, giving advantages over the bloodstream [5]. Besides these considerations, metastatic processes are usually supported by a significant increase in the formation of new lymphatic vessels, named lymphangiogenesis, in the primary tumors and in the regional draining lymph nodes (LNs) [6].

In clinical practice, special attention is paid to the regional LNs as the main players in the metastatic dissemination [7]. Thus, LN status (presence or absence of tumor cells) is used as a potential diagnostic marker for predicting the pathologic stage of the disease, and it is essential for therapeutic strategy decisions [8]. It has been reported that tumor-draining LNs in cancer patients show enhanced lymphangiogenesis even before of metastatic colonization [9, 10]. LNs may serve as a permissive pre-metastatic lymphvascular niche providing a supportive environment for the survival and proliferation of metastatic cells and promoting their further movement to distal organs [10]. Currently, breast cancer patients treated with hormonal or anti-angiogenic therapies combined with other agents are suffering from recurrence of secondary tumors in draining LNs [11, 12]. Inhibition of angiogenesis results in hypoxic condition in tumors that provokes the overexpression of lymphangiogenic factors, enhancing tumor metastasis through lymphatics [13, 14]. Therefore, targeting lymphangiogenesis represents a potential strategy to prevent or treat lymphatic metastases. However, only few drugs designed for the blocking of this crucial event are in clinical trials nowadays (Tivantinib, Onartuzumab, Rilotumumab, Trebananib, and IMC-3C5) [8, 15]. Most of these anti-lymphangiogenic compounds are drugs targeting the VEGF-C/VEGFR-3 signaling axis, the most relevant and specific pathway that promotes lymphangiogenesis in pathological situations [15].

In our continuous efforts to discover and characterize new anti-angiogenic compounds, we previously screened a plethora of natural compounds. AD0157, a pyrrolidinedione isolated from the fermentation broth of the marine fungus *Paraconiothyrium* sp. HL-78-gCHSP3-B005, was found to be the more potent anti-angiogenic drug [16]. On the basis of these findings, we sought to determine its anti-tumor and, especially its anti-lymphangiogenic properties. Herein, we report for the first time that in the treatment of human breast cancer xenografts in mice, AD0157 reduces tumor growth, blocks the invasion of tumor cells to the draining LNs, and potently reduces metastases, through a strong reduction of the lymphatic vasculature in both primary tumors and in regional LNs. Evidences supporting AD0157 as an anti-lymphagiogenic drug include the inhibitory biologic effects of this compound in a wide experimental battery of in vivo, ex vivo, and in vitro models. AD0157 also induces apoptosis in lymphatic endothelial cells (LECs) and mechanistically blocks VEGFR-3/-2 signaling pathways. Altogether, our results shed light on the promising therapeutic potential of AD0157 as a new anti-lymphangiogenic and anti-tumor drug in the treatment of lymphatic metastases.

## Methods

### Drug preparation

AD0157 compound (Additional file 1: Figure S1) obtained from Biomar Institute S.A (León, Spain) was dissolved in DMSO and stored in frozen aliquots until use. DMSO was used in controls at the same percentage used in the experimental conditions (up to 0.1%). For all assays, a pilot study was first conducted to optimize the range of the more effective AD0157 concentrations.

### Animals

NOD/SCID mice, C57BL/6 mice, and Wistar rats were purchased from Charles River (Saint-Germain-Nuelles, France). Animal care and experimental procedures were performed in strict compliance with the European Communities Council Directive 2010/63/EU and the Belgium legislation for the animal experimentation. All experimental protocols were approved by the Local Animal Ethics Committee at the University of Liège (13/1522), and the 3Rs principles were always implemented.

### Cell culture and transfection

MDA-MB-231 breast adenocarcinoma cells were obtained from the ATCC, and MDA-MB-231 cells expressing luciferase (MDA-MB-231/Luc+) were generated by transfection with a plasmid containing the luciferase reporter (Lipofectamine/Plus Reagent, Invitrogen). They were grown in DMEM supplemented with glucose (4.5 g/L), glutamine (2 mM), penicillin (50 IU/mL), streptomycin (50 mg/L), amphotericin (1.25 mg/L), and 10% FBS, at 37 °C with 5% CO_2_ in air, until reaching 80% of confluency. LECs used in this study were from adult human dermal lymphatic microvasculature (hMVEC.dLy.Ad) and were purchased from Lonza. LECs were cultured in complete endothelial growth microvascular medium (EGM-2 medium), composed of EBM-2 and single quotes, including 0.2% (*v*/*v*) hydrocortisone, 2% (*v*/*v*) hFGF-B, 0.5% (*v*/*v*) VEGF, 0.5% (*v*/*v*) R3-IGF-1, 0.5% (*v*/*v*) hEGF, 0.5% (*v*/*v*) ascorbic acid, 0.5% (*v*/*v*) Gentamicin/Amphotericin-1000, and 5% (*v*/*v*) FBS, at 37 °C and humidified 5% CO_2_ atmosphere, until reaching 90–100% of confluency. All experiments were carried out with LECs of less than five passages.

### Mice experiments for toxicology

NOD/SCID mice (*n* = 3) were daily treated for 30 days with intraperitoneal injections of the maximal AD0157 dose (3 mg/kg) used in the in vivo tests. According to the ethical protocol approved by the Local Animal Ethics Committee, the appearance, behavior, body weight, motility, eating and drinking habits, skin turgor, and urine output of mice were daily inspected to detect signs of toxicity, pain, or distress. Moreover, after mice sacrifice, the internal organs were inspected to ensure the absence of inflammation, hemorrhage, or necrosis, among others.

### Orthotopic mammary fat pad tumor growth in mice

MDA-MB-231/Luc+ cell suspensions (2 × 10^6^ cells in 50:50 DPBS/Matrigel) were injected subcutaneously into the fourth abdominal mammary glands of female NOD/SCID mice. Tumor growth was assessed by measuring the length and width of tumors every 3–4 days (tumor volume = length × width^2^ × 0.4) [17]. Mice bearing tumors with 50–60 mm^3^ (day 20) were randomized into different groups and treated daily with either vehicle (saline solution), 1.5 mg/kg or 3 mg/kg AD0157 drug. For in vivo imaging, mice were intraperitoneally injected with 75 mg/kg D-luciferin and the Lumina II IVIS instrument (Caliper Life Sciences) was used for bioluminescence measurement according to manufacturer’s recommendations. Animals were sacrificed when tumor volume exceeded 600 mm^3^, and tumors were harvested, weighed, and subjected to immunohistochemistry or quantitative RT-PCR analyses. Axillary LNs and the main mouse organs were excised, the ex vivo bioluminescent signals were measured, and they were preserved for immunohistological or quantitative RT-PCR analyses.

### Immunohistochemistry

Mammary tumors, LNs, and the main mouse organs were harvested, fixed, dehydrated, embedded in paraffin and sectioned in 5-μm slides. Then, samples were deparaffined, hydrated, and autoclaved for 11 min at 126 °C in Target Retrieval Solution (Dako). Endogenous peroxidase activity was quenched (3% H_2_O_2_ in PBS), and sections were blocked. For lymphatic vasculature detection, a primary polyclonal LYVE-1 antibody was used (1/100, R&D Systems) and samples were revealed with the Phenol Red chromogen kit (Dako). To detect MDA-MB-231/Luc+ cells, a mouse monoclonal anti-human-ki-67 antibody (1/100, clone MIB-1, M7240, Dako) was applied and the signal was developed by treatment with 3,3’-diaminobenzidine (DAB, Dako). Finally, samples were counterstained with hematoxylin/eosin, washed, dehydrated, mounted, and visualized.

### Quantitation of gene expression

RNA was extracted from mammary tumors, LNs, and LECs using the RNeasy Mini kit (Qiagen). Tumors and LNs were previously frozen and pulverized with MagNA Lyser (Roche), and reverse transcription was conducted on 1 μg of total RNA (First Strand cDNA Synthesis Kit, Roche) followed by real-time PCR (FastStart SYBR Green Master, Roche) with the following specific primers (Eurogentec): sense, 5′- TCCTGGTATGACAATGAATACGG-3′, and antisense, 5′- TCTCTTGCTCAGTGTCCTTGCT-3′, for GADPH; sense, 5′-CCTCGTGCAAGACCTTTCCATT-3′, and antisense, 5′-CCCACACCTGGGGTTTGAGAAA-3′, for LYVE-1; sense, 5′-CCCACGCAGACATCAAGACG-3′, and antisense, 5′-TGCAGAACTCCACGATCAGC-5′, for VEGFR-3; and sense, 5′-TTCCACGTGACCAGGGGTCCT-3′, and antisense, 5′-AGCTGCCTGACCACGCAATGT-3′, for VEGFR-2. Quantification was performed by normalization of the values obtained for the endogenous GADPH rRNA amplification.

### In vivo lymphangiogenesis assays

#### Mouse corneal neovascularization assay

Inflammatory corneal neovascularization was induced by thermal cauterization (Optemp II V; Alcon Surgical) in the central cornea of anesthetized C57BL6 mice [18]. Next, intraperitoneal injections with vehicle (saline solution) or AD0157 (1.5 or 3 mg/kg) were daily administered during 8 days. At mice sacrifice, corneas were dissected, fixed, blocked, and double immunostained for lymphatic and blood vessel detection, as detailed previously [18]. Lymphatic and blood vasculatures were quantified with the toolbox of MATLAB 8.3 (R2014a) software, and the following parameters were analyzed: area, branching (number of bifurcations), end-point (number of sprout tips) and length densities, and the number and length of filopodias [19].

#### Mouse ear sponge assay

Sterile compressed gelatin sponges (Gelfoam, Pfizer) were cut in small cylindrical fragments (~3 mm^3^) and incubated with serum-free DMEM containing recombinant human (rh) VEGF-C (1 μg/mL; R&D Systems) and with or without AD0157. Then, they were soaked with interstitial type I collagen gel and implanted into the mouse ears. Every 2 days, serum-free DMEM containing AD0157 or not (controls) were injected in the apex of the ear, and after 3 weeks, the ears were excised and frozen in tissue optimal cutting temperature (OCT) compound (VWR Chemical). Blocks were sectioned, processed for lymphatic and blood vessel immunodetection, scanned, and automatically quantified, as previously described [20].

### Ex vivo lymphangiogenesis approaches

#### Three-dimensional mouse lymphatic ring explants

The lymphatic sprouting from explants was analyzed using ex vivo mouse 3D-lymphatic ring cultures [21]. Briefly, thoracic ducts dissected from C57BL6 mice were cut into 1-mm pieces and embedded in rat tail interstitial type I collagen gel. Explants were cultured in MCDB131 (Invitrogen) supplemented with 2% Ultroser G (Pall Life Sciences), in the presence or absence of AD0157, at 37 °C in 5% O_2_, 5% CO_2,_ and 90% N_2_ for 7 days. Cultures were photographed, and computerized quantifications were performed on binary images. A grid of concentric rings was generated by successive increments at fixed intervals of thoracic duct boundary, and the number of microvessel-grid intersections (N_i_) was counted [21].

#### Rat mesentery cultures

Mesenteric windows, the translucent and thin connective tissue between artery/vein pairs in the small intestine, were surgically dissected from adult Wistar rats (Charles River), as described [22]. Explants were cultured in serum-free MEM supplemented with rhVEGF-C (200 ng/mL), with or without AD0157 for 5 days. Whole mounted explants were washed, fixed, permeabilized, and immunolabeled with an anti-VEGFR-3 primary antibody (1/50; Santa Cruz Biotechnology) and an Alexa Fluor 488-conjugated secondary antibody (1/200; Invitrogen). Rat mesenteric windows were visualized, and computerized analyses were performed to analyze the lymphangiogenic response.

### In vitro lymphangiogenesis tests

#### Cell proliferation assay

The 3-(4,5-dimethylthiazol-2-yl)-2,5-diphenyltetrazolium bromide or MTT dye reduction assay in 96-well microplates was used [20]. Briefly, LECs (3 × 10^3^ cells/well) and MDA-MB-231/Luc+ cells (2 × 10^3^ cells/well) were incubated with serial dilutions of AD0157 for 3 days, and then, MTT (5 mg/mL in PBS) was added. IC_50_ values were calculated as those concentrations of AD0157 yielding 50% cell survival, taking the values obtained for control as 100%.

#### Tubulogenesis assay

LECs (5 × 10^5^ cells/well) were embedded in a collagen matrix containing or not AD0157 and cultured in 2% FBS supplemented EGM-2 medium, with or without the drug. The formation of capillary-like structures was monitored in the next 24 h, and pictures were quantified with the image analysis toolbox of MATLAB 8.3 (R2014a) software (Mathworks, Inc).

#### Migration and invasion assays

The migratory activity was assessed using the scratch assay. Cells in a confluent monolayer were scratched and supplied with complete medium containing 2% FBS, in the absence or presence of AD0157. Wounded areas were photographed at 0 and 48 h of incubation. Mitomycin C (0.1 μg/ml; Sigma-Aldrich) was added to inhibit cellular proliferation. The percentage of recovered area was determined by image analysis (NIH Image 1.6 software). For invasion assays, LECs (1.5 × 10^5^) in EBM-2 medium containing 0.5% FBS, with or without AD0157, were seeded in the upper compartment of Transwell inserts (Corning) coated with 0.2% gelatin. The lower compartment was filled with EBM-2 containing 1% FBS and rhVEGF-C (400 ng/ml; R&D Systems). After 48 h, cells were fixed, stained with Giemsa solution (Millipore), and filters were visualized and quantified.

#### Spheroid assay

LEC spheroids were generated as previously described [23], embedded in collagen gels with or without AD0157 and cultured in 2% FBS supplemented EGM-2 medium for 24 h. Then, spheroids were examined and pictures were analyzed using a computer-assisted method of quantification [24]. The convex envelope area (minimal convex polygon area containing the spheroid core and all sprouting cells), the migrated LEC area (area containing migrating cells), and the LEC density (number of pixels belonging to cells that intersect the circle “i”, *N*_i_, normalized by the corresponding perimeter *P*_i_) with the maximal length (Lmax) were analyzed.

### Apoptosis and cell cycle analyses

Cells were treated or not with AD0157 during 14 h, and apoptosis was evaluated by Hoechst 33258 staining, flow cytometry, and caspase-3-7 activity. For Hoechst staining, cells were fixed, stained with Hoechst 33258 (1 μg/mL, Sigma-Aldrich), and observed under a fluorescence microscope (Leica, TCS-NT). For cell cycle analysis, cells were fixed, stained with propidium iodide solution (40 μg/mL propidium iodide and 0.1 mg/mL RNase-A; Sigma-Aldrich) and percentages of subG1, G1, and S/G2/M populations were determined using a MoFlo Dakocytomation cytometer (Dako, Denmark). For the determination of caspase-3/-7 activity, the Caspase-Glo® 3/7 reagent, provided in the ApoTox-GloTM Triplex Assay Kit (Promega), was used according to manufacturer’s instructions.

### Immunoblotting

Serum-starved subconfluent LEC cultures were incubated in the presence or absence of AD0157 for 2 h and then challenged for 30 additional minutes with rhVEGF-C (400 ng/mL), rhVEGF-C156S (500 ng/mL; R&D Systems), or rhVEGF-A (100 ng/mL; R&D Systems). Cell lysates were analyzed by SDS-PAGE, electrotransferred to nitrocellulose membranes (GE Healthcare Life Sciences), and blots were probed with primary antibodies against pVEGFR-3 (1/1000; Cell Application), VEGFR-3 (1/1000; Millipore), pVEGFR-2, VEGFR-2, pERK1/2, ERK1/2, pAkt, Akt, (1/1000; Cell Signaling), and GADPH (1/2000; Millipore). Detection was carried out with chemiluminescence system *ECL Western Blotting Substrate* (Pierce), and bands were quantified and expressed as phosphorylated protein/total protein ratio.

### Statistical analysis

Statistical analysis was performed using GraphPad Prism 5.0 software (San Diego, CA, USA). For the tumor growth and metastasis incidence, one-way ANOVA and chi-square tests were applied, respectively. Otherwise, results were analyzed using the non-parametric Mann-Whitney test; *p* < 0.05 was considered significant. All data are expressed as means ± s.e.m. (standard error of the mean).

## Results

### AD0157 inhibits tumor growth and tumor-associated lymphangiogenesis in orthotopic mammary xenografts

Human breast adenocarcinoma MDA-MB-231/Luc+ cells were injected into the fourth mammary glands of NOD/SCID mice, and tumor growth was continuously monitored. In mice administrated with the higher AD0157 dose (3 mg/kg), tumor growth was drastically blocked after 10 days of the first drug injection, with the maintenance of this inhibitory pattern until the end of the experiment (Fig. 1a). AD0157 did not exhibit any toxicity assessed by mice body weight measurements (Fig. 1b), visual examinations, and inspection of the internal organs at sacrifice. IVIS imaging and bioluminescence quantifications at the end of the experiment revealed smaller tumor sizes in AD0157-treated mice. Furthermore, the tumor-inhibitory effect of AD0157 was more potent in those mice injected with 3 mg/kg than in the group injected with 1.5 mg/kg (Fig. 1c, d). Tumor weight of harvested mammary tumors (Fig. 1e) and macroscopic photographs (Fig. 1f) further confirmed that AD0157 significantly decreased the MDA-MB-231/Luc+ xenograft growth.

**Fig. 1:** AD0157 reduces tumor growth and lymphangiogenesis in orthotopic mammary xenografts. **a** Evolution of tumor volumes in NOD/SCID mice implanted with MDA-MB-231/Luc+ cells and treated daily with vehicle (saline solution) or AD0157 (1.5 or 3 mg/kg) for 25 days, as indicated on top of the graph. *Dashed line* indicates the tumor volume (50 mm^3^) reached by tumors before drug treatment. *Crosswise lines* indicate the starting point for the statistical differences shown at right. **b** Mouse body weights before and during treatments. *ns* denotes no statistical differences between groups. **c** Representative in vivo bioluminescent signals of mice at the end of the treatment. **d** Quantification of tumor bioluminescent radiance. **e** Tumor weights at the end of the experiment. **f** Representative pictures of tumors harvested from mice treated with vehicle (control) or AD0157 (1.5 and 3 mg/kg). Each square represents a surface of 2.25 cm^2^. **g** Representative histological sections showing human ki-67 (proliferation marker, in *brown*) and LYVE-1 (lymphatic vessel marker, in *dark pink*) stainings in mammary tumors. *Scale bars* represent 100 μm. **h** Quantification of human ki-67^+^ cell and lymphatic densities in histological sections of mammary tumors. Data are presented as mean ± s.e.m. One-way ANOVA significance test, followed by the Bonferroni test, was used to compare the tumor growth in the different conditions. The Wilcoxon-Mann-Whitney was applied for the rest of statistical tests. *p < 0.05, **p < 0.01, ***p < 0.001 (*n* = 12 mice/group)

To examine tumor cell proliferation and tumor-associated lymphangiogenesis in primary tumors, immunohistochemical analyses were performed. Treatments with AD0157 decreased the density of human proliferating cells (Ki-67^+^ cells) and the density of lymphatic vasculature in tumors (Fig. 1g). A 1.7 and 2.4-fold decrease in Ki-67^+^ cell density was seen in mice treated with 1.5 and 3 mg/kg AD0157, respectively (0.36 ± 0.017 versus 0.25 ± 0.021, *p* < 0.05; 0.36 ± 0.017 versus 0.15 ± 0.018, *p* < 0.001). Importantly, a potent anti-lymphangiogenic effect of this compound was shown by the huge reduction of the lymphatic density upon treatment: 2.2 and 9-fold reduction with 1.5 and 3 mg/kg AD0157, respectively (0.09 ± 0.008 versus 0.04 ± 0.006, *p* < 0.001; 0.09 ± 0.008 versus 0.01 ± 0.002, *p* < 0.001) (Fig. 1h). These data were confirmed by analyzing the messenger RNA (mRNA) expression of LYVE-1 in complete mammary tumors extracts (Additional file 2: Figure S2).

### AD0157 reduces tumor colonization and lymphatic density in draining LNs

Tumor-draining LNs from MDA-MB-231/Luc+ tumor-bearing mice were resected after mice sacrifice. Control groups frequently developed tumor-draining LN metastases, with 100% of LNs positive for bioluminescent signal (presence of tumor cells) (Fig. 2a). In contrast, only 65 and 30% of the analyzed LNs showed positivity for the presence of human breast cancer cells, in mice daily treated with 1.5 and 3 mg/kg AD0157, respectively (Fig. 2a). In addition, LNs harvested from AD0157-treated mice were smaller than those belonging to control ones (Fig. 2a). Quantification of the ex vivo bioluminescent signals through Xenogen acquisitions revealed a significant decrease in the averaged bioluminescence of tumor-draining LNs from AD0157-treated mice (Fig. 2b). These data were confirmed by a clear reduction in the Ki-67^+^ cell density in LNs (Fig. 2c, d). Interestingly, the maximal distance (Lmax) reached by tumor cells inside the LNs (distance measured from the LN edge) was drastically decreased (Fig. 2d). In addition, tumor-draining LNs harvested from control mice displayed enlarged lymphatic vessels, and they were distributed throughout the paracortex and medullar area, reaching values of 0.1 ± 0.007 for the lymphatic density and 0.47 for the Lmax (Fig. 2c, d). In sharp contrast, LNs from mice injected with 3 mg/kg AD0157 showed a lower lymphatic density (0.048 ± 0.01) together with a diminished Lmax (0.31), being the lymphatic vasculature mostly located in the paracortical region (Fig. 2c, d). LYVE-1 mRNA expression in complete LNs validated the previous results (Additional file 2: Figure S2). These data clearly indicate that AD0157 blocks LN colonization as well as lymphatic vasculature remodeling in draining LNs.

**Fig. 2:** AD0157 reduces tumor colonization and lymphatic density in draining LNs. **a** Representative pictures of ex vivo bioluminescent signals recorded in draining LNs at mice sacrifice. The percentage of positive LNs for tumor cells is indicated. **b** Quantification of bioluminescent radiance in LNs. **c** Immunostainings of human Ki-67 (proliferative cells in *brown*, *left panels*) and LYVE-1 (lymphatic vessels in *dark pink*, *right panels*) in whole LN histological sections. Panels at high magnification illustrate the region delineated by the *square* in the complete LNs. *Scale bars* represent 250 μm. **d** Human ki-67^+^ cell density (surface occupied by tumor cells divided by the total LN surface), lymphatic density (surface occupied by lymphatic vessels divided by the total LN surface), and spatial distributions of tumor cells and lymphatic vessels in LNs. The spatial distribution is calculated from the LN edge, where the distance is equal to 0

### AD0157 potently prevents metastases in distant organs

To determine whether AD0157 could prevent tumor cell invasion and distant metastases, the main organs (brain, lungs, intestines, kidneys, spleen, and uterus) were resected at mice sacrifice and examined with the IVIS imaging system. The organs from mice injected with the saline solution (drug vehicle) exhibited higher bioluminescent signals compared to those organs resected from mice treated with AD0157, indicating an anti-metastatic effect of this drug (Fig. 3a). Immunostainings for human Ki-67 confirmed the presence of infiltrating tumor cells in the different organs (Fig. 3b). AD0157 treatment (1.5 and 3 mg/kg) prevented the development of distant metastases (Fig. 3c). Interestingly, only the liver in one mouse (8.3%) and the lungs in two mice (16.7%) showed tumor cells in mice treated with 3 mg/kg AD0157, and no metastatic dissemination was found in the rest of the analyzed organs (Fig. 3c).

**Fig. 3:** AD0157 prevents distant metastases. **a** Representative ex vivo bioluminescent signals of distant organs (brain, lungs, liver, intestines, kidneys, spleen, and uterus). **b** Immunohistochemical images visualizing micrometastases by human Ki-67 detection (in *brown*). *Scale bars* represent 250 μm. **c** Number and percentage of organs colonized by metastatic cells. Data are presented as mean ± s.e.m., and the Wilcoxon-Mann-Whitney significance tests were used to compare the differences between vehicle (control) and AD0157 treatment. Chi-square with Yates’ correction test was used to analyze the metastasis incidence. *p < 0.05, **p < 0.01, ***p < 0.001 (*n* = 12 mice/group)

To determine whether tumor cells and LECs were equally sensitive to this drug, MDA-MB-231/Luc+ cells and LECs were subjected in vitro to different AD0157 concentrations for IC_50_ value calculations. LEC proliferation was suppressed with at least 5- fold lower dose than MDA-MB-231/Luc+ one (IC_50_ = 2.5 μM for LECs and IC_50_ = 13.8 μM for MDA-MB-231/Luc+) (Additional file 3: Figure S3). These data suggested that LECs were the most susceptible to AD0157 and prompted us to apply the drug in different in vivo and ex vivo lymphangiogenesis models.

### AD0157 impairs pathological lymphangiogenesis in vivo and interferes with the lymphangiogenic process ex vivo

We further explored the efficacy of AD0157 in inhibiting lymphangiogenesis in vivo and ex vivo. In an inflammatory mouse corneal model, although at day 9 post-injury, lymphatic vasculature was evident in mice treated with the vehicle, AD0157-treated mice exhibited a reduced lymphatic vascular network (Fig. 4a). Computerized quantifications revealed a decrease in the length and end-point lymphatic densities in corneas of mice treated with 1.5 and 3 mg/kg AD0157. Furthermore, the lymphatic area and branching densities were diminished in corneas of mice administered with the highest AD0157 dose (3 mg/kg/day) (Fig. 4b). The spatial distribution curve of lymphatic vessels around the limbus revealed impaired migration of vessels towards corneal center in AD0157-treated mice (Fig. 4b). We next analyzed the migrating cells at the tip of the lymphatic buds, characterized by numerous cytoplasmic extensions or filopodias. A decrease in the number and length of filopodia-like extensions was found in corneas of treated mice (Fig. 4a, b). On the other hand, the ear sponge assay revealed that sponges soaked with rhVEGF-C and AD0157 at different concentrations displayed decreased lymphatic vessel density (Fig. 5a, b). Importantly, the highest dose of AD0157 (2.5 nmol) drastically suppressed the lymphangiogenic response with a 5-fold reduction compared with untreated and rhVEGF-C-stimulated sponges (Fig. 5b). Furthermore, in this experimental condition most lymphatic vessels remained located close to the sponge border, with a maximal distance of lymphatic vessel penetration (Lmax) of 1.3 mm, while in rhVEGF-C-stimulated sponges lymphatic vessels reached a distance superior of 1.7 mm (Fig. 5b).

**Fig. 4:** AD0157 impairs corneal neovascularization in mice. **a** Representative flat-mounted cauterized corneas harvested from control and AD0157-treated mice at day 9 post-injury. Lymphatic (LYVE-1 positive) and blood (CD31 positive) vessels appear in *green* and in *red*, respectively, at low (*left panels*) and high (*middle panels*) magnifications. *Scale bars* represent 1000 and 500 μm, respectively. Panels at right correspond to representative pictures of filopodia-like structures (*white arrowheads*) displayed by migrating LECs. *Scale bars* represent 10 μm. **b** Computerized measurements of different parameters: lymphatic area density (area covered by neoformed lymphatic vessels), length density (cumulative length of vessels), branching density (number of bifurcations), end-point density (number of sprout tips), spatial lymphatic distribution (a grid was applied on each cornea picture to establish the distribution curves of capillaries around the limbal vessels; N_i_ corresponds to the number of vessel intersections with the grid *versus* the distance to the limbus), number and length of filopodia-like structures in a total length of 25 μm at the end of the lymphatic vessel, and blood area density (area covered by neoformed blood vessels). Results were divided by the total cornea area to obtain densities. Values are expressed as mean ± s.e.m., and the Wilcoxon-Mann-Whitney significance tests were used to compare the differences between control and AD0157 treatments.*p < 0.05, **p < 0.01, ***p < 0.001 (*n* = 12 mice/group)

**Fig. 5:** AD0157 inhibits in vivo VEGF-C-induced lymphangiogenesis and blocks the lymphangiogenic process ex vivo. **a** Representative pictures of gelatin sponges soaked with either rhVEGF-C (1 μg/mL) alone (positive control) or rhVEGF-C + AD0157 at different concentrations and implanted between the mouse ear skin layers. Lymphatic and blood vasculatures were examined by LYVE-1 (*green*) and CD31 (*red*) immunostainings, respectively. Dapi staining was used to detect cell nuclei (*blue*). *Scale bars* represent 1500 and 500 μm on higher magnification. A total of 10 mice were analyzed in each experimental condition. **b** The graphs represent the computerized quantification of the lymphatic density (*left panel*), the normalized frequency of lymphatic vessels from the sponge edge to its center (*middle panel*), and the blood density (*right panel*). *Arrows* indicate the maximal distance of LEC migration (Lmax). **c** Ex vivo lymphatic sprouting from mouse thoracic duct explants embedded in a type I collagen gel and cultured in the absence (control) or presence of AD0157 for 7 days. *Scale bars* represent 500 μm. **d** *Graphs* represent the number of microvessel intersections (N_i_) quantified on binarized images using a grid of concentric rings (*left graph*) and the LEC density at a distance (*d*) = 0.25 mm from the ring border (*right graph*). A total of 10 lymphatic rings collected from five different mice were analyzed in each experimental condition. **e** Microvessel outgrowth in rat mesenteric windows incubated in medium containing either rhVEGF-C (200 ng/mL) alone or in combination with AD0157, ranging from 0.5 to 2.5 μM, for 5 days. *Scale bars* represent 200 μm. **f** Lymphatic density and number of branchings in rat mesenteric windows exposed or not to AD0157. A total of 10 mesenteric windows harvested from five different rats were evaluated in each experimental condition. Values are expressed as mean ± s.e.m., and the Wilcoxon-Mann-Whitney significance tests were used to compare the differences between control and AD0157 treatment. *p < 0.05, **p < 0.01, ***p < 0.001

As the two above-described lymphangiogenesis models are also suitable for investigating angiogenesis, the impact of the studied drug on the blood network was evaluated in corneas and mouse ear sponges. As expected, the highest concentration of AD0157 (3 mg/kg) induced a reduction in blood vessel formation (Figs. 4 and 5a, b). These data are in line with our previous work about the anti-angiogenic properties of AD0157 [16]. Interestingly, AD0157 was more potent on lymphangiogenesis than on angiogenesis, and doses able to interfere with the lymphangiogenic process were not potent enough to block the angiogenic one (Figs. 4b and 5b).

Ex vivo cell sprouting and outgrowing of new lymphatic endothelial capillaries was evaluated in lymphatic rings [21] cultured with or without different doses of AD0157. While control explants exhibited an important lymphatic outgrowth at day 7, AD0157 decreased the number of microvessels and fully blocked LEC sprouting upon 2.5 μM (Fig. 5c, d). To further validate these results, the drug was added to rat mesenteric windows incubated in the presence of rhVEGF-C (200 ng/mL). AD0157 at 2.5 μM reduced to half the lymphatic vessel density and the number of branchings (Fig. 5e, f).

### AD0157 blocks tube formation, migration, invasion, and sprouting of LECs in vitro

To investigate how AD0157 affects the lymphangiogenic process, a battery of in vitro assays was used. Again, a dose-dependent effect of AD0157 was observed in all the models, with a drastic blockade in the studied LEC property when the drug was used at 1 μM. Thus, the compound impaired the organization of LECs in a 3D-network of tubes with a reduction in the tube area density and the number of branchings (Fig. 6a, b). In the wound-healing assay (Fig. 6c, d) and in Boyden chambers (Fig. 6e, f), AD0157 inhibited the migration and invasion of LECs. Moreover, AD0157 treatment blocked vessel sprouting in the LEC spheroid model, which mimic the 3D environment in which LECs proliferate, migrate, and form new tubes (Fig. 6g). A huge reduction of LEC sprouting and migration was achieved at AD0157 1 μM as assessed by the different parameters measured: (i) the convex envelop area; (ii) the area occupied by migrated cells; (iii) the spatial distribution of sprouting cells around the spheroid core, and, finally, (iv) the cell density at a distance of 0.13 mm of the spheroid center (Fig. 6h). Surprisingly, doses of AD0157 up to 10 μM were needed to interfere with MDA-MB-231/Luc+ cell migration in the scratch assay (Additional file 4: Figure S4a, b).

**Fig. 6:** AD0157 suppresses lymphangiogenesis in vitro by interfering with LEC tubulogenesis, migration, invasion, and sprouting. **a** Tube-like structures formed by LECs in a collagen matrix, in the absence (control) or presence of different AD0157 concentrations. *Scale bars* represent 200 μm. **b** Computerized quantification of the tube area density and the number of branchings (common point between 2 or more tubes). **c** Pictures showing the area recovered by LECs after 48 h of wounded LEC monolayers, in the absence or presence of different AD0157 doses. *Dashed lines* in pictures indicate the initial (time 0) wound edges. *Scale bars* represent 100 μm. **d** Percentage of the initial cell-free area recovered by endothelial cells. **e** Representative images of the invaded LECs across a Transwell chamber coated with 0.2% gelatin, after 48 h of treatment. **f** Percentage of invaded cells. **g** LEC sprouting from spheroids embedded in a collagen-methyl cellulose gel under different experimental conditions. *Scale bars* represent 100 μm. **h** Computerized quantifications of the convex envelope area (minimal convex polygon area containing the spheroid core and all sprouting cells), the migrated cell area (area containing migrating cells), the LEC density (number of pixels belonging to cells that intersect the circle “i”, N_i_, normalized by the corresponding perimeter) at different distances from the spheroid core and values of the LEC density at the specific distance of 0.13 mm from the spheroid centre, in control and AD0157-treated spheroids. *Arrows* indicate the maximal length (Lmax). Values are expressed as mean ± s.e.m., and the Wilcoxon-Mann-Whitney significance tests were used to compare the differences between control and AD0157 treatment. *p < 0.05, **p < 0.01, ***p < 0.001 (*n* = 5 independent tests)

### AD0157 induces LEC apoptosis

Firstly, chromatin morphology was analyzed in treated and untreated cells stained with Hoechst 33258 (Fig. 7a). AD0157 provoked chromatin condensation at 0.5 and 1 μM in 21.3 and 29.5% of cells, respectively (Fig. 7b). To confirm this finding, cell cycle analyses by flow cytometry were performed in LECs stained with propidium iodide. In Fig. 7c are displayed representative flow cytometry diagrams showing increased apoptotic subG1 cell subpopulation upon AD0157 treatment. AD0157 used at 0.5 and 1 μM led to a 5- to 6-fold enhancement of apoptotic cells (Fig. 7d). It is worth mentioning that differences were detected not only in the subG1 but also in the S/G2/M subpopulations (Fig. 7d). Moreover, the “effector” caspase-3/-7 activity, which plays a crucial role in the apoptosis induction, was activated upon AD0157 treatment (0.5 and 1 μM) (Fig. 7e). Importantly, AD0157 was more potent to induce LEC apoptosis than MDA-MB-231/Luc+ cell apoptosis, and higher drug concentrations were required to obtain similar effects in breast cancer cells (Additional file 4: Figure S4c-e).

**Fig. 7:** AD0157 induces apoptosis in LECs. Analysis of apoptosis in LECs treated or not with AD0157 for 14 h. **a** Chromatin condensation revealed by Hoechst 33258 staining. *Scale bars* represent 100 μm. **b** Percentages of cells with condensed chromatin (total cells were counted by using bright field). **c** Cell cycle distribution in LECs stained with propidium iodide and analyzed by flow cytometry. **d** Percentages of subG1 (apoptotic cells with invariable DNA content), G1 (cells in interphase before cell division), and S/G2/M (DNA replication and mitosis) LEC subpopulations. **e** LEC Caspase-3/-7 activity. Values are expressed as mean ± s.e.m., and the Wilcoxon-Mann-Whitney significance tests were used to compare the differences between control and AD0157 treatment. *p < 0.05, **p < 0.01, ***p < 0.001 (*n* = 5 independent tests)

### AD0157 interferes with the activation of VEGFR-3, VEGFR-2, and downstream mediators

Since VEGFR-2, and especially VEGFR-3, are expressed in LECs and involved in lymphangiogenesis, we first investigated whether AD0157 could modulate the expression levels of both receptors. However, VEGFR-3 and VEGFR-2 mRNA levels were similar in the absence or presence of this compound (Fig. 8a). It is also well known that activation of VEGFR-3/2 heterodimers and/or VEGFR-3 homodimers through phosphorylation mainly triggers the lymphangiogenic response [25]. Herein, LECs were stimulated with different growth factors (rhVEGF-C, rhVEGF-C156S, or rhVEGF-A). Stimulation with rhVEGF-C resulted in VEGFR-3 activation, as well as stimulation with rhVEGF-A led to a VEGFR-2 induction (Fig. 8b). Downstream actors such as ERK1/2 and Akt were also activated after growth factor addition (Fig. 8b). Interestingly, a pretreatment with AD0157 at 0.5 and 1 μM decreased VEGFR-3, VEGFR-2, ERK1/2, and Akt phosphorylation levels (Fig. 8b, c). Similarly, VEGFR-3, ERK, and Akt activations were obtained after stimulation with rhVEGF-C156S, a mutant rhVEGF-C form, which binds VEGFR-3, but not VEGFR-2. In this experimental situation, only the higher AD0157 dose (1 μM) was able to inhibit VEGFR-3 and downstream mediator phosphorylations (Fig. 8b, c). Therefore, AD0157 exerts, at least in part, its inhibitory function through an interference with the VEGFR-3 and VEGFR-2 signaling pathway activations.

**Fig. 8:** AD0157 blocks VEGFR-3 and VEGFR-2 signaling cascades in LECs. **a** Values of VEGFR-3 and VEGFR-2 mRNA expression levels in LECs incubated with different AD0157 concentrations. **b** Representative Western-blots showing the effect of AD0157 on VEGFR-3, VEGFR-2, ERK1/2, and Akt phosphorylations after stimulation with rhVEGF-C (400 ng/mL), rhVEGF-C156S (500 ng/mL), or rhVEGF-A (100 ng/m). **c** Quantification by densitometry of Western blots. Results are expressed as the percentage of phosphorylated proteins/total protein ± s.e.m. of five Western blots. The Mann-Whitney-Wilcoxon test was used to determine if the differences among control (stimulated LECs without AD0157 treatment) and AD0157-treated and stimulated LECs were statistically significant. *p < 0.05, **p < 0.01, ***p < 0.001 versus control

## Discussion

In this work, we are assigning unprecedented and very potent anti-lymphangiogenic and anti-local and distant metastatic functions to a natural compound, AD0157. For the preclinical characterization of AD0157 as a powerful lymphangiogenic inhibitor, a panel of 3 in vivo, 2 ex vivo, and 7 in vitro models has been applied. We have first used the mammary fat pad xenograft model, which recapitulates human breast cancer growth and metastatic dissemination to regional LNs and distant organs, including the brain, lungs, and liver, as observed in patients. MDA-MB-231/Luc+ breast cancer cells used in this approach highly express VEGF-C, the main lymphangiogenic factor promoting VEGFR-3 activation leading to tumor-associated lymphangiogenesis [26–29]. Our results demonstrate that mammary tumors markedly regressed under AD0157 treatment and lymphatic vessel formation was inhibited in these primary tumors. Importantly, the impaired lymphatic vessel formation induced by AD0157 within primary tumors was associated with reduced metastasis in draining LNs. Moreover, given that the incidence of the organ metastasis was also reduced by AD0157 treatment, restricting metastasis to regional LNs by AD0157 could be useful to suppress systemic dissemination of breast cancer cells.

Next, to determine the respective properties of AD0157 on LECs and cancer cells, we investigated in vitro the effect of this drug on LECs and MDA-MB-231/Luc+ cell proliferation. Interestingly, LECs showed a substantially lower IC_50_ value than MDA-MB-231/Luc+ cells with this agent. Moreover, this value was also lower than those already described for other endothelial cells and tumor cells [16], revealing that LECs were the most sensitive cells to the studied drug. In line with the above consideration, it is worth noting that AD0157 blocked MDA-MB-231/Luc+ migration at 5 μM but not at the lower doses (≤1 μM) used for LECs. This assumption was further supported by the higher doses needed to induce apoptosis on MDA-MB-231/Luc+ cells, compared with the apoptotic induction achieved by AD0157 on LECs. Moreover, the IC_50_ value for LECs was lower than that observed in other endothelial cells [16]. All these findings provided an evidence-based reason for the rational in-depth characterization of AD0157 in different in vivo, ex vivo, and in vitro lymphangiogenesis models. In all models used, a dose-response inhibition was observed in the lymphatic growth, migration, sprouting, and tubulogenesis. Therefore, the compound is able to interfere with the different main steps of the lymphangiogenic process. Besides its anti-lymphangiogenic properties, the apoptosis induction by AD0157 can be considered as an additional ability supporting the mechanism of lymphangiogenesis suppression and may contribute to the effectiveness of the drug. Collectively, these data emphasize the powerful anti-lymphangiogenic activity of AD0157, which is reinforced in vivo by the effect, although less efficient, exerted on tumor cells. They underline the multifactorial feature of this natural compound without any obvious systemic toxic effects.

From a mechanistic standpoint, we demonstrated that AD0157 is a dual inhibitor. Treatment with this drug abrogated the activation of VEGFR-2, and especially of VEGFR-3, induced by rhVEGF-A and rhVEGF-C or VEGF-C156S, respectively. VEGFR-3 plays a pivotal role in the lymphatic vascular formation, and VEGFR-3 inhibition has been shown to disrupt the cellular functions of LECs and adult lymphangiogenesis [5]. On the other hand, VEGFR-2 could be involved in lymphangiogenesis through its indirect effect on LECs by forming heterodimers with VEGFR-3 [5]. Moreover, phosphorylations of downstream molecules such as ERK and Akt were suppressed upon AD0157 treatment as well. Given the recognized crucial roles played by ERK- and Akt-dependent signaling cascades in the development of many tumors types and resistance to chemotherapy [30, 31], this AD0157 property should be taken into account for further therapeutic evaluations.

Targeting VEGF and VEGFR signaling in a tumor has been considered as a promising and attractive therapeutic strategy, and several approaches have been investigated, including the use of antibodies against VEGF receptors [32, 33], small tyrosine kinase inhibitors [34–36], and soluble receptors that trap lymph/angiogenic factors [37]. For instance, targeting the VEGF pathway in gastric cancers has gained increasing attention after the results obtained in phase III clinical trials, which demonstrate superior survival outcome with some anti-angiogenic drugs, such as ramucirumab, apatinib, and bevacizumab, than with the standard therapy [38]. Nevertheless, further studies are required to deeply explore the timing and potentially predictive biomarkers of angiogenesis inhibitors to improve the selection of patients and improve clinical benefit. Other tyrosine kinase inhibitors are displaying interesting properties in the clinic. Anlotinib, a broad-spectrum anti-tumor drug designed to primarily inhibit VEGFR2/3, FGFR1-4, PDGFR α/β, c-Kit, and Ret, has shown manageable toxicity, long circulation, and anti-tumor potential in patients with advanced refractory solid tumors in phase I clinical trials [39].

Given the complexity and redundancy of the VEGF signaling network in promoting angiogenesis and lymphangiogenesis, multitargeting by small molecules may be an appropriate strategy for effective inhibition of tumor-associated lymphangiogenesis. The suppression of either VEGFR-3 or VEGFR-2 alone might not be sufficient to inhibit cellular signaling and the whole lymphatic process. AD0157 has been reported as an anti-angiogenic drug in different models: the chicken chorioallantoic membrane assay (CAM), the intersegmental vessel formation in transgenic TG(fli1:EGFP)y1 zebrafish embryos, the aortic ring assay, and a battery of in vitro tests [16]. The superior potency of AD0157 against lymphangiogenesis over angiogenesis is here supported in two additional pathological models of angio/lymphangiogenesis, the corneal model and the ear sponge assay.

From a clinical perspective, it is worth mentioning that the tyrosine kinase inhibitor sunitinib, available for the treatment of renal cell carcinoma and metastatic gastrointestinal stromal tumors that prove resistant to imatinib [40–42], has been used in our laboratory in the MDA-MB-231/Luc+ xenograft and in the mouse cornea models [17, 18]. Long-term treatment with sunitinib at a therapeutic dose of 40 mg/kg for 30 days resulted in a drastic inhibition of primary tumor growth, metastasis formation, and corneal lymphangiogenesis [17, 18]. In both in vivo approaches, sunitinib was used at 40 mg/kg/day, while treatments with 3 mg/kg/day AD0157 have shown similar inhibitory effects in the same models. These observations reflect that AD0157 is a potent compound and might be of benefit in the treatment of cancer by suppressing lymphangiogenesis and LN metastasis. In addition, this study also highlights the absence of toxicity in mice during AD0157 treatment, a fact that can help in the challenge of predicting toxicity in patients based on preclinical models. All together demonstrate the interest of considering this compound for future clinical investigations.

Finally, and perhaps most importantly, this timely study provides an example of how primary tumors are tightly connected with their local microenvironment and sheds light on the important role played by the lymphatic vasculature in cancer progression. Therefore, using multifunctional compounds such as AD0157, displaying anti-lymphangiogenic, anti-angiogenic, and anti-tumoral properties, is a very promising strategy to counteract cancer progression and metastatic dissemination.

## Conclusions

Here, we assign uncovered and potent in vivo, ex vivo, and in vitro anti-lymphangiogenic functions to AD0157. This drug through its dual VEGFR-3 and VEGFR-2 cascades inhibition and its apoptotic effect blocks lymphangiogenesis and prevents LN and distant metastases in a breast cancer model. Our results demonstrate the interest of considering this compound for future clinical investigations. The efficacy of AD0157 in other tumor cell types and mouse models will be explored in future approaches. Hopefully, this study can also serve as a precedent for applying similar therapeutic strategies in lymphatic metastases chemoprevention.

## Additional files

Additional file 1: Figure S1. Chemical structure of AD0157. (PS 139 kb)

Additional file 2: Figure S2. AD0157 reduces LYVE-1 mRNA expression in mammary tumors and in draining LNs. Analyses of LYVE-1 expression by qRT-PCR, normalized to GADPH expression, in mammary MDA-MB-231/Luc+ tumors and LNs resected from control and AD0157-treated mice. Values are expressed as mean ± s.e.m. and Wilcoxon-Mann-Whitney significance tests were used to compare the differences between control and AD0157 treatments. *p < 0.05, **p < 0.01, ***p < 0.001 (*n* = 12). (PS 296 kb)

Additional file 3: Figure S3. AD0157 inhibits LEC and MDA-MB-231/Luc+ cell proliferation. Representative curves showing the dose-dependent effect of AD0157 on the in vitro growth of LEC and MDA-MB-231/Luc+ cells. Cell proliferation is represented as a percentage of untreated cells. Each point represents the mean of quadruplicates; SD values were typically lower than 10% of the mean values and are omitted for clarity. The half-maximal inhibitory concentration (IC_50_) value was calculated from dose-response curves as the concentration of compound yielding 50% of control cell survival. It is expressed as means ± s.e.m. of five independent experiments. (PS 415 kb)

Additional file 4: Figure S4. Effect of AD0157 on MDA-MB-231/Luc+ cell migration and apoptosis. (a) Closure of the initial scratched area by MDA-MB-231/Luc+ cells after 48 h in the absence or presence of different AD0157 doses. Broken lines in pictures indicate the initial (time 0) wound edges. Scale bars represent 100 μm. (b) Graph shows the percentage of the initial cell-free area recovered by tumor cells. (c) Representative pictures showing the effect of AD0157 on MDA-MB-231/Luc+ cell chromatin condensation after 14 h of treatment. Scale bars represent 100 μm. (d) Percentages of control and AD0157-treated tumor cells with condensed chromatin (total cells were counted by using bright field). (e) Percentages of subG1, G1, and S/G2/M MDA-MB-231/Luc+ cell subpopulations analyzed by flow cytometry after AD0157 treatment. (PS 17413 kb)

## Abbreviations

ERK: Extracellular signal regulated kinases
LECs: Lymphatic endothelial cells
LNs: Lymph nodes
LYVE-1: Lymphatic vessel endothelial hyaluronan receptor 1
MTT: 3-(4,5-Dimethylthiazol-2-yl)-2,5-diphenyltetrazolium bromide
VEGFR: Vascular endothelial growth factor receptor
